This article has been retracted.

# HOXA7 plays a critical role in metastasis of liver cancer associated with activation of *Snail*

**DOI:** 10.1186/s12943-016-0540-4

**Published:** 2016-09-06

**Authors:** Bo Tang, Guangying Qi, Xiaoyu Sun, Fang Tang, Shengguang Yuan, Zhenran Wang, Xingsi Liang, Bo Li, Shuiping Yu, Jie Liu, Qi Huang, Yangchao Wei, Run Zhai, Biao Lei, Xinjin Guo, Songqing He

**Affiliations:** 1 Department of Hepatobiliary Surgery, Guilin Medical University, Affiliated Hospital, Guilin, 541001 Guangxi People’s Republic of China; 2 Laboratory of Liver Injury and Repair Molecular Medicine, Guilin Medical University, Guilin, 541001 Guangxi People’s Republic of China; 3 Department of Pathology and Physiopathology, Guilin Medical University, Guilin, 541004 Guangxi People’s Republic of China; 4 Department of Gastroenterology, First Affiliated Hospital of Dalian Medical University, Dalian, 116011 Liaoning People’s Republic of China; 5 Department of Clinical Pharmacology, College of Pharmacy, Dalian Medical University, Dalian, 116011 Liaoning People’s Republic of China

**Keywords:** HOXA7, Metastasis, Liver cancer, Snail

## Abstract

**Background:**

Liver cancer is one of the main causes of cancer-related death in human. HOXA7 has been proved to be related with several cancers.

**Method:**

The expression levels of HOXA7 were examined by Western blot, qRT-PCR or ICH. MTT was used to detect the proliferative rate of liver cancer cells. The invasive abilities were examined by matrigel and transwell assay. The metastatic abilities of liver cancer cells were revealed in BALB/c nude mice.

**Results:**

In this report, we revealed that HOXA7 promoted metastasis of HCC patients. First, increased levels of HOXA7 were examined in liver cancer especially in metastatic liver cancer. Moreover, higher expression level of HOXA7 was associated with poorer prognosis of liver cancer patients. Overexpression of HOXA7 significantly enhanced proliferation, migration, invasion in vitro and tumor growth and metastasis in vivo meanwhile silencing HOXA7 significantly inhibited the aboves abilities of liver cancer cells. In this research, we identified that HOXA7 performed its oncogenic characteristics through activating *Snail*.

**Conclusion:**

Collectively, we identify the critical role and possible mechanism of HOXA7 in metastasis of liver cancer which suggest that HOXA7 may be a potential therapeutic target of liver cancer patients.

**Electronic supplementary material:**

The online version of this article (doi:10.1186/s12943-016-0540-4) contains supplementary material, which is available to authorized users.

## Background

Liver cancer is one of the leading causes of cancer-related death all around the world [1, 2]. In recent years, significant advances in diagnosis and treatment of liver cancer are reported, but unfortunately, patients with liver cancer still have a very dismal long-term prognosis. In clinic, partial liver resection is the treatment of choice for liver cancer patients [3]. However, intrahepatic recurrence and metastasis which simultaneously predict poor outcome are the main challenges in the treatment of patients with liver cancer. The identification of critical biomarkers that suppress or promote these processes may lead to novel therapeutic targets for improving the prognosis of these patients.

As shown in reports, epithelial to mesenchymal transition (EMT), a phenomenon observed in developmental program, is evoked during tumor invasion and metastasis [4]. Researchers have discovered several molecular pathways that mediate EMT in cancers [5–8]. EMT could promote tumor cell invasion and metastasis as well as lead to the generation of cancer stem cells with increased self-renewal and tumor-initiating capabilities and increased resistance to apoptosis and chemotherapy [4, 9]. During EMT, dynamic changes in gene expression and cytoskeletal re-organization are often discovered [10]. One of the significant changes is loss of E-cadherin which is essential for cell to cell adhesion, and suppression of E-cadherin is one of the key steps in EMT which not only disrupts cell to cell adhesions but also promotes cellular invasion and metastasis [11].

Science researchers have revealed that EMT is closely related with multiple regulatory networks containing signaling pathways [12] and transcription factors [13]. Among them, Zinc finger protein Snail is mostly reported to be associated with EMT and metastasis [14]. Snail, as a transcription factor, could bind to E-box sequences located in the promoter regions of target genes activation of which could induce EMT and promote cell invasion and metastasis [15].

In this study, we detected that the expression levels of Snail and EMT markers were regulated by Homeobox protein A7 (HOXA7) which belong the *HOX* gene family. Homeodomain-containing transcription factors encoded by this gene were known to be key regulators of embryonic development [16]. Moreover, HOXA7 has been reported to be associated with progression of some tumors [17]. Here we explored the possible mechanism of EMT activated by HOXA7 in the metastasis of liver cancer.

## Methods

### Clinical samples and cell culture

Samples of liver cancer and their adjacent tissue samples are obtained from the First Affiliated Hospital of Dalian Medical University. For survival analysis, the essential information of the liver cancer patients was collected from the First Affiliated Hospital of Dalian Medical University. Parts of the samples are frozen in liquid nitrogen for RNA or protein examination and the other parts are fixed in paraformaldehyde for immunohistochemistry. All cell lines are cultured in adaptive culture medium according to ATCC and cultured at 37 °C in 5 % CO2.

### Establishment of cell lines

Human gene *HOXA7* was cloned into pBabe-puro vector and shRNA of *HOXA7* and *Snail* were cloned into pSuper-puro vector. Retrovirus supernatants of containing pBabe, pSuper, pBabe-HOXA7, pSuper-shHOXA7 #1, pSuper-shHOXA7 #2 and pSuper-shSnail were produced in Phoenix packaging cells. We respectively transfected indicated cell lines with these different viral supernatant containing 4 μg/ml polybrene (Sigma). Then cells were selected by puromycin (2 μg/ml).

### RNA extraction, reverse transcription, and real-time RT-PCR

Total RNA was extracted from freshly-frozen samples or cells with TRIzol reagent (Invitrogen). Total RNA was reverse-transcribed with First Strand cDNA Synthesis Kit (Invitrogen). Real time PCR reactions were conducted using Platinum SYBR Green qPCR SuperMix-UDG reagents (Invitrogen) on the PRISM 7900HT system (Applied Biosystems). All reactions were done in triplicate and reactions without reverse transcriptase were used as negative controls. The GAPDH were used as the endogenous controls and the 2-ΔΔCT equation was used to calculate the relative expression levels.

### Western blot analysis

Western blot analysis was conducted using anti-HOXA7, anti-Snail, anti-E-cadherin, anti-N-cadherin, anti-α-catenin, anti-vimentin and anti-β-actin. All antibodies were purchased from Cell Signaling Technology.

### Proliferation assay

MTT (3-[4, 5-dimethylthiazol-2-yl]-2, 5-diphenyl-tetrazolium bromide, Solarbio, M8180) assay were used to detect the proliferative rate of indicated cell lines. 1000 cells were plated into 96-well plate and cultured at 37 °C. MTT was dropped at 70 % density and the 96-well plate was incubated for 4 h followed 150 μl DMSO dropped after removing the supernatant carefully. The OD values were measured by the machine (Multiskan 3) at 0, 24, 48 and 72 h.

### Transwell and matrigel assay

The effects of HOXA7 or Snail expression on cell migration and invasion were assessed using the wound-healing and Transwell assays as previously described [18].

### Immunohistochemical analysis

Following deparaffinization, liver cancer sections were immunohistochemically analyzed using antibodies for HOXA7, respectively, and subsequently were pathologically confirmed for the tumor phenotype and specific immunostaining. The positive cells were counted under a microscope and analyzed.

### In vivo tumor growth model

Male BALB/c nude mice aged 4 to 6 weeks were purchased from the Hunan Slac Jingda Laboratory Animal Co., Ltd (Changsha, China). For tumor growth assay, indicated cells were resuspended in PBS and 3 × 10^6^ cells (200 μl) were subcutaneously injected in the axilla of nude mice. Six weeks later, mice were sacrificed, and tumors were dissected and weighted. Animal handling and research protocols were approved by the Animal Care and Use Ethnic Committee.

### In vivo metastasis

Male BALB/c nude mice aged 4 to 6 weeks were purchased from the Hunan Slac Jingda Laboratory Animal Co., Ltd (Changsha, China). For metastasis assay, cells were resuspended in PBS at a concentration of 3 × 10^7^ cells/ml. Cell suspension (0.1 ml) was injected into tail veins of nude mice. All of the mice were killed by CO_2_ 60 days after inoculation.

### Chromatin immunoprecipitation (ChIP)-qPCR

ChIP kit was purchased from Millipore and ChIP experiments were carried out essentially as described [19]. Immnuoprecipitated DNA was analyzed on the ABI PRISM 7900HT sequence detection system. The primers used for detection of promoters after ChIP are available upon request.

### Luciferase reporter assays

The cDNA encoding HOXA7 was subcloned into the expression vector pBabe and subcloning was confirmed with sequencing by Shanghai Genechem Co., Ltd. The pGL3 reporter construct plasmid (−3000/+100) consisted of a 3100-bp genomic DNA fragment of the Snail promoter (Promega, Madison, WI, USA). The pGL3-Snail promoter plasmid or its negative control pGL3-basic plasmid carrying the firefly luciferase reporter were co-transfected with an internal control, pRL-TK Renilla vector (Promega), by using Lipofectamine 2000 (Invitrogen). In addition, cells were respectively transfected with 600 ng of HOXA7 overexpression plasmid pBabe or its negative control pbabe-vector. Cell lysates were harvested 48 h after transfection. The firefly and renilla activities were measured by the Dual-Luciferase Reporter Assay System (Promega). Firefly luciferase activity was normalized to the Renilla luciferase activity. Each transfection was repeated three times.

### Statistical analysis

Statistical analysis Data were described as the mean ± SD. Survival analysis was estimated using the Kaplan–Meier method. The relationship between survival period and each of the variables was analyzed using the log-rank test for categorical variables. Comparisons between different groups were undertaken using the Student two-tailed *t* test. The criterion of statistical significance was *P* < 0.05. Statistical analysis was done with SPSS/Win11.0 software (SPSS Inc.).

## Results

### Ectopic levels of HOXA7 are related with metastasis and prognosis of liver cancer

At the first time, we confirmed whether HOXA7 expression level was elevated in liver cancer by western blot. As shown in Additional file 1: Figure S1A, the expression of HOXA7 was significantly increased in tumors. Moreover, HOXA7 was overexpressed in 73.85 % liver cancer samples (48 samples of total 65 samples). Then we analyzed the relationship between HOXA7 and metastasis and found that both mRNA level (Fig. 1b) and protein levels (Additional file 1: Figure S1B) of HOXA7 was significantly elevated in metastatic liver tumors. Moreover, the increased protein level of HOXA7 was confirmed in 9 pairs of liver cancer samples (Fig. 1c). These results above revealed that elevated level of HOXA7 was possibly correlated with metastasis of liver cancer.

**Fig. 1:** The expression of HOXA7 is increased in metastatic liver cancer. **a** Quantification of *HOXA7* in liver cancer samples. **b** Analysis of *HOXA7* levels in non-metastatic and metastatic liver cancer tissues. Non-metastatic: cancer tissues without metastasis; metastatic: cancer tissues with metastasis. **c** Western Blot analysis of HOXA7 levels in some liver cancer samples. *P* < 0.01 in panel b based on the Student *t* test. *Error bars*, SD. The each number of replicates is 3

In order to further confirm the role of HOXA1 in liver cancer, we identified HOXA7 expression level in tumor samples. As shown in Fig. 2a, different expression levels of HOXA7 were found in tumor sections by immunochemical stain. Quantificational analysis showed that positive expression of HOXA7 was examined in 89 % tumor tissues (Fig. 2b) while negative expression of HOXA7 was examined in 88 % noncancerous tissues (Fig. 2c). Then we confirmed whether HOXA7 was related with prognosis of liver cancer patients, we carried out the bioinformatics analysis of the dataset of liver cancer patients. As shown in Fig. 2d, positive levels of HOXA7 were significantly related with poorer survival of liver cancer patients compared with those with negative HOXA7 expression suggesting that HOXA7 was correlated with prognosis of liver cancer patients.

**Fig. 2:** HOXA7 is overexpressed and related to the prognosis of liver cancer patients. **a** Immunohistochemical analysis of HOXA7 levels in liver cancer tissues and normal liver tissues. **b** Proportion analysis of HOXA7 levels in liver cancer tissues. **c** Proportion analysis of HOXA7 levels in normal liver tissues. **d** Survival analysis of patients with liver cancers in an available dataset. The each number of replicates is 3

### HOXA7 accelerates liver cancer cell migration and invasion

To better understand the role of HOXA7 in liver cancer, we first examined HOXA7 levels in liver cancer cell lines (Fig. 3a and b), then we used retroviral vectors to establish liver cancer cell lines stably overexpressing or silencing HOXA7. The expression levels of HOXA7 in the subsequent cell lines were examined by Western blotting (Fig. 3c and e) and qRT-PCR (Fig. 3d and f). We next examined the effects of HOXA7 on migration and invasion of liver cancer cells. Transwell and matrigel assay revealed that silencing HOXA7 significantly inhibited MHCC97H (Fig. 4a and b) and HCCLM3 (Additional file 2: Figure S2A and B) migrated or invaded through the membrane to the bottom of the aperture while overexpression of HOXA7 promote these progresses in HeG2 (Fig. 4c and d) and HL-7702 (Additional file 3: Figure S3A and B). These results revealed that HOXA7 promotes migration and invasion of liver cancer cells.

**Fig. 3:** Examination of HOXA7 levels in established cell lines. **a** Western Blot analysis of HOXA7 levels in liver cancer cell lines. **b** qRT-PCR analysis of *HOXA7* levels in liver cancer cell lines. **c** Western Blot analysis of HOXA7 levels in MHCC97H and HCCLM3 cells silencing HOXA7. **d** qRT-PCR analysis of *HOXA7* levels in MHCC97H and HCCLM3 cells silencing HOXA7. **e** Western Blot analysis of HOXA7 levels in HepG2 and HL-7702 cells overexpressing HOXA7. **f** qRT-PCR analysis of *HOXA7* levels in HepG2 and HL-7702 cells overexpressing HOXA7. *P* < 0.01 in panel b, d and f based on the Student *t* test. *Error bars*, SD. The each number of replicates is 3

**Fig. 4:** HOXA7 promotes migration and invasion of liver cancer cells. **a** MHCC97H silencing HOXA7 possessed less migrating and invading abilities in traswell and martigel assay. **b** The migrated or invaded cells silencing HOXA7 were plotted as the average number of cells in five random fields. **c** HepG2 overexpressing HOXA7 possessed more migrating and invading abilities in traswell and martigel assay. **d** The migrated or invaded cells overexpressing HOXA7 were plotted as the average number of cells in five random fields. *P* < 0.01 in panel b and d based on the Student *t* test. *Error bars*, SD. The each number of replicates is 3

### HOXA7 acts oncogenic properties in vivo

To further confirm whether HOXA7 promote metastasis in vivo, MHCC97H cell silencing HOXA7 or HepG2 cell overexpressing HOXA7 were inoculated into tail vein of BALB/C athymic mice respectively. Eight weeks later, we observed that less mice injected with MHCC97H cell silencing HOXA7 had distant metastasis (Fig. 5a). Moreover, less metastatic foci in lung (Fig. 5c and d) were counted in each mouse injected with liver cancer cell silencing HOXA7. On the contrary, overexpressing HOXA7 significantly increased the number of metastatic mice (Fig. 5b) and metastatic foci in lung (Fig. 5e and f).

**Fig. 5:** HOXA7 promotes metastasis of liver cancer. **a** The total numbers of mice with distant metastasis at 60 days after injection of MHCC97H cells with silent expression of HOXA7 into tail vein. **b** The total numbers of mice with distant metastasis at 60 days after injection of HepG2 cells with ectopic expression of HOXA7 into tail vein. **c** HE stain for metastatic foci in lung with injection of MHCC97H cell silencing HOXA7. **d** The number of metastatic foci in lung with injection of MHCC97H cell silencing HOXA7. **e** HE stain for metastatic foci in lung with injection of HepG2 cell overexpressing HOXA7. **f** The number of metastatic foci in lung with injection of HepG2 cell overexpressing HOXA7. *P* < 0.01 in panel d and f based on the Student *t* test. *Error bars*, SD. The each number of replicates is 3

On the other hand, the effects of HOXA7 on cell proliferation and tumor growth were examined by MTT and tumor formation assay. As shown in Additional file 4: Figure S4A, silencing HOXA7 significantly inhibited cell proliferation of liver cancer cells while overexpressing HOXA7 promoted this progress (Additional file 4: Figure S4B). Tests in vivo revealed that silencing HOXA7 significantly supressed tumor growth in vivo and induced a decrease in tumor weights (Additional file 4: Figure S4C). In contrast, overexpression of HOXA7 accelerated tumor growth and induced an increase in tumor weights (Additional file 4: Figure S4D). Tests in vivo revealed that HOXA7 could promote tumor growth and metastasis of liver cancer.

### Snail is essential for HOXA7-induced metastasis

HOXA7 was proved to be related with metastasis of liver cancer above. To better understand the mechanisms by which HOXA7 engaged in metastasis, we performed gene expression profiling on MHCC97H-shHOXA7 and its control cells. Microarray analysis identified numbers of genes significantly differentially expressed after silencing HOXA7 (Fig. 6a) and Snail targets were the top related genes (Fig. 6b). We next examined Snail expression levels in liver cancer cells overexpressing or silencing HOXA7. As shown in Fig. 7a, decreased expression levels of Snail were identified in liver cancer cells silencing HOXA7 by western blot (Fig. 7a) and qRT-PCR (Fig. 7b). In contrast, increased expression levels of Snail were found in liver cancer cells overexpressing HOXA7 by western blot (Fig. 7c) and qRT-PCR (Fig. 7d). To further confirm whether Snail was regulated by HOXA7, we use linear correlation analysis to verify the relationship between HOXA7 and Snail. As shown in Fig. 7e, the expression levels of Snail were positively correlated with the expression levels of HOXA7. Moreover, we examined expression levels of Snail targets. As shown in Additional file 5: Figure S5A, silencing HOXA7 significantly increased epithelial cell markers (E-cadherin and α-catenin) and decreased mesenchymal cell markers (N-cadherin and vimentin) while overexpression of HOXA7 showed the opposite effects (Additional file 5: Figure S5B). The similar changes in EMT markers were confirmed by qRT-PCR (Additional file 5: Figure S5C, D, E and F).

**Fig. 6:** HOXA7 is related with Snail. **a** Supervised hierarchical clustering of the genes differentially expressed after silent expression of PKM2. **b** Gene set enrichment analysis was carried out using ConceptGen. Snail is the top related gene of HOXA7

**Fig. 7:** HOXA7 elevates expression level of Snail. **a** Western blot analysis of Snail in liver cancer cells with silencing HOXA7. **b** qRT-PCR analysis of *Snail* in liver cancer cells with silencing HOXA7. **c** Western blot analysis of Snail in liver cancer cells with overexpression of HOXA7. **d** qRT-PCR analysis of *Snail* in liver cancer cells with overexpression of HOXA7. **e** Linear correlation analysis between Snail and HOXA7. *P* < 0.01 in panel b and d based on the Student *t* test. *Error bars*, SD. The each number of replicates is 3

To study the mechanism by which HOXA7 activated Snail, we performed quantitative chromatin immunoprecipitation (qChIP) assay in liver cancer cells with silence or overexpression of HOXA7. We found that silencing HOXA7 was associated with decreased *Snail* levels at region -2400-2150 in MHCC97H (Fig. 8b) and HCCLM3 (Fig. 8c). More occupancy of those *Snail* gene promoter regions by HOXA7 was detected in HepG2-HOXA7 (Fig. 8d) and KL-7702-HOXA7 (Fig. 8e). Moreover, in order to validate the binding relationship between HOXA7 and the promoter of Snail, we performed luciferase reporter asssay, as shown in Additional file 6: Figure S6, HOXA7 significantly increased the activity of Snail promoter. These results clearly indicated that HOXA7 induces transcriptional activation of *Snail* by regulating promoter of *Snail*.

**Fig. 8:** HOXA7 combines to the promoter of *Snail*. **a** Schematic presentation of two regions relative to the *Snail* transcriptional start site used as primers to test HOXA7 occupied abundance. **b** and **c** qChIP was performed to assess HOXA7 occupancy in liver cancer cells with silent expression of HOXA7. IgG was used as negative control. **d** and **e** qChIP was performed to assess HOXA7 occupancy in liver cancer cells with overexpression of HOXA7. IgG was used as negative control. *P* < 0.01 in panel b-e based on the Student *t* test. *Error bars*, SD. The each number of replicates is 3

In order to confirm whether Snail was essential for HOXA7-induced metastasis, we silenced Snail in liver cancer cells with overexpression of HOXA7. Expression levels of Snail were examined by western blot (Fig. 9a) and qRT-PCR (Fig. 9b). We found that silencing Snail significantly inhibited the numbers of cells migrated or invaded through the membrane to the bottom of the aperture of HepG2-HOXA7 cell (Fig. 9c) and KL-7702-HOXA7 cell (Fig. 9d).

**Fig. 9:** Snail is essential for HOXA-induced metastasis. **a** Western blot analysis of Snail in indicated cell lines. **b** qRT-PCR analysis of *Snail* in indicated cell lines. **c** Transwell and matrigel assay of HepG2-HOXA7 cell with silent expression of Snail. **d** Transwell and matrigel assay of HL-7702-HOXA7 cell with silent expression of Snail. **e** The total numbers of mice with distant metastasis at 60 days after injection of HepG2-HOXA7 cells with silent expression of Snail into tail vein. **f** HE stain for metastatic foci in lung with injection of HepG2-HOXA7 cell with silent expression of Snail. **g** Numbers of metastatic foci in lung with injection of HepG2-HOXA7 cell with silent expression of Snail. **h** Conclusion of regulatory mechanism of HOXA7 in this study. *P* < 0.01 based on the Student *t* test. *Error bars*, SD. The each number of replicates is 3

Collectively, HOXA7 activates Snail expression by combining to the promoter of *Snail*. And increased target proteins of Snail promote the metastasis of liver cancer. In a word, Snail is essential for the HOXA7-induced metastasis.

## Discussion

Homeobox genes were first identified in the fruit fly *Drosophila melanogaster* [20]. 39 HOX genes locating on different chromosomes numbered from 1 to 13 and are organized into four clusters labeled A, B, C and D [21]. In this study, we investigated the expression, function, and mechanisms of HOXA7 in liver cancer. We found that HOXA7 expression is elevated in liver cancer and higher level of HOXA7 is associated with poorer prognosis of liver cancer patients. Liver cancer cells with higher expression of HOXA7 were more aggressive and mesenchynal. Overexpression of HOXA7 significantly promotes cell proliferation, migration and invasion in vitro and tumor growth and metastasis in vivo. Of note, we revealed that HOXA7 activates *Snail* expression by combining to the promoter of *Snail* which may be the mechanism of HOXA7-induced invasion and metastasis (Fig. 9h).

The HOX family is critical for various aspects of differentiation and morphogenesis both in the embryo and in adult tissues [22]. Recently, an increasing number of studies have indicated that HOX genes play important roles in oncogenesis [23–25]. Many cancers exhibit altered HOX gene expression, particularly leukemia, breast, prostate and lung carcinomas [26–30]. It has been reported that HOXA7 stimulates human hepatocellular carcinoma proliferation through cyclin E1/CDK2 [25]. However, the specific functional role of HOXA7 in liver cancer remains unclear. We here revealed that HOXA7 promotes metastasis of liver cancer and the liver cancer patients with high HOXA7 level have a dismal long-term prognosis. Moreover we revealed the mechanism of HOXA7-induced metastasis correlated with snail. These findings point out a novel regulatory network of metastasis in liver cancer.

Metastasis is considered to be the main cause of cancer-related death, and EMT is proved to be the key step of metastasis [31, 32]. In reports, EMT can be induced by transcription factor Snail [33] which is a repressor of E-cadherin gene expression [15]. Moreover, loss of E-cadherin has been considered to be one hallmark of EMT [34]. Snail, as the main regulatory of E-cadherin, has been discussed in multiple papers. In this study, we revealed a novel regulator of Snail. HOXA7 could directly activate gene expression of *Snail* and induced EMT in liver cancer cells which could improve the Snail-related networks. HOXA7, as an upstream regulator of Snail, may be a novel therapeutic and prognostic target of liver cancer.

## Conclusions

In summary, high level of HOXA7 was related with poorer prognosis of liver cancer patients. Overexpression of HOXA7 significantly promoted invasion and metastasis of liver cancer cells by activating Snail expression suggesting that HOXA7 may be a novel therapeutic and prognostic target of liver cancer.

## Additional files

Additional file 1: Figure S1. Ectopic HOXA7 expression was related with metastasis of liver cancer. (A) Analysis of HOXA7 levels in noncancerous and tumorous tissues. (B) Analysis of HOXA7 levels in non-metastatic and metastatic liver cancer tissues. *P* < 0.01 in panel A and B based on the Student *t* test. Error bars, SD. The each number of replicates is 3. (JPG 976 kb) Additional file 2: Figure S2. Silencing HOXA7 inhibits migration and invasion of HCCLM3 cell. (A) HCCLM3 silencing HOXA7 possessed less migrating and invading abilities in traswell and martigel assay. (B) The migrated or invaded cells silencing HOXA7 were plotted as the average number of cells in five random fields. *P* < 0.01 in panel B based on the Student *t* test. Error bars, SD. The each number of replicates is 3. (JPG 1592 kb) Additional file 3: Figure S3. Overexpression of HOXA7 promotes migration and invasion of HL-7702 cell. (A) HL-7702 with overexpression of HOXA7 possessed more migrating and invading abilities in traswell and martigel assay. (B) The migrated or invaded cells overexpressing HOXA7 were plotted as the average number of cells in five random fields. *P* < 0.01 in panel B based on the Student *t* test. Error bars, SD. The each number of replicates is 3. (JPG 1188 kb) Additional file 4: Figure S4. HOXA7 promotes cell proliferation and tumor growth of liver cancer cell. (A) MTT assay of liver cancer cells with silent expression of HOXA7. (B) MTT assay of liver cancer cells with overexpression of HOXA7. (C) Tumor formation assay of liver cancer cells with silent expression of HOXA7. (D) Tumor formation assay of liver cancer cells with overexpression of HOXA7. ***P* < 0.01 based on the Student *t* test. Error bars, SD. The each number of replicates is 3. (JPG 3241 kb) Additional file 5: Figure S5. HOXA7 promotes expression levels of EMT markers. (A) Western blot analysis of EMT markers in liver cancer cells with silent expression of HOXA7. (B) Western blot analysis of EMT markers in liver cancer cells with overexpression of HOXA7. (C) qRT-PCR analysis of EMT markers in liver cancer cells with silent expression of HOXA7. (D) qRT-PCR analysis of EMT markers in liver cancer cells with overexpression of HOXA7. *P* < 0.01 in panel C-F based on the Student *t* test. Error bars, SD. The each number of replicates is 3. (JPG 4138 kb) Additional file 6: Figure S6. Lucifease reporter assay show that HOXA7 significantly increases the activity of the prromoter of Snail. (JPG 266 kb)
